The article "An Optimized Decision Method for Smart Teaching Effect Based on Cloud Computing and Deep Learning" was retracted in 2023. Reasons: signs of a paper mill; suspected computer-generated content; unreliable results or conclusions; lack of ethics approval or compliance.

# An Optimized Decision Method for Smart Teaching Effect Based on Cloud Computing and Deep Learning

**DOI:** 10.1155/2022/6907172

**Published:** 2022-03-26

**Authors:** Miaomiao Jiang, Yuwei Sun

**Affiliations:** Physical Education College of Harbin University of Commerce, Harbin 150028, China

## Abstract

In order to improve the effect of intelligent teaching and give full play to the role of intelligent technology in modern physical education, in this paper, cloud computing and deep learning methods are used to comprehensively evaluate the teaching effect of colleges and universities, and calculate the evaluation effect and accuracy. Cloud computing and deep learning algorithm combine the teaching evaluation scale, teaching content, and characteristics to formulate teaching plans for different students and realize targeted teaching evaluation. The results show that the teaching evaluation method proposed in this paper can improve students' learning interest by about 30%, enhance learning initiative by about 20%, and the matching rate between the actual teaching effect and the expected requirements is 98%. Therefore, cloud computing and deep learning model can improve the accuracy of teaching effect evaluation in colleges and universities, provide support for the formulation of teaching evaluation schemes, and promote the development of intelligent teaching in colleges and universities.

## 1. Introduction

Cloud computing and deep learning was first applied in the field of power and gradually developed to the field of teaching in the later stage. Cloud computing and deep learning can have a key impact on the improvement of students' learning status and teaching content, and improve the overall teaching effect. In 2017, China Education Commission put forward the strategy of “comprehensive quality education” and the concept of “double reduction,” which reduced the college tennis teaching time from 48 hours in 2012 to 32 hours in 2020, with a decrease of 30% [1]. The results are shown in Figure 1. In this paper, tennis intelligent teaching is taken as an example to analyze the advanced nature and intelligent advantages of intelligent teaching. At the same time, the increase of multimedia, online teaching, and practical courses also greatly reduces the teaching hours of college tennis physical education. With the continuous reduction of teaching hours, the teaching pressure of tennis teachers is increasing and even affects the effect of classroom teaching. Therefore, “teaching optimization of cloud computing and deep learning” has been put on the agenda [2] and has become the research focus of tennis teaching in major universities. Cloud computing is the mainstream algorithm at present. Through the intelligent search of the data in the network, the horizontal teaching effect evaluation can be realized. Deep learning is the in-depth study of teaching contents and methods to realize the vertical analysis of teaching effect. The integration of cloud computing and deep learning can realize the comprehensive analysis of intelligent teaching and improve the accuracy of effect evaluation. Although cloud computing and deep learning methods are traditional teaching evaluation methods, this paper integrates the two and constructs a new theoretical model, which belongs to a new model attempt. The advantage of the first mock exam is very obvious. It can not only expand the scope of the evaluation of the intelligent teaching effect but also increase the depth of assessment and effectively remedy the deficiency of the single model. Foreign scholars began to study cloud computing and deep learning in 2010, and gradually introduced it into the evaluation of intelligent teaching effect. At the same time, foreign countries have achieved good research results in data preprocessing in cloud computing and data mining in deep learning. However, there is a gap between China and foreign countries in terms of intelligent devices and development procedures. Moreover, the national conditions and policies of foreign countries are different from those at home, so it is impossible to copy them. Therefore, domestic scholars should strengthen the research of cloud computing and deep learning, and integrate it with intelligent teaching.

At present, tennis teaching mainly adopts the form of “unified“ teaching, which has the advantages of unified teaching content and simple teaching methods, but it cannot meet the “personalized” requirements of students [3]. Under the background of reducing teaching time, increasing teaching pressure, and improving the requirements of quality education, there will be problems of reduced interest in learning and lack of learning law. On this basis, this paper proposes a cloud computing and deep learning model to integrate students' learning data, classify students' interests, and analyze the learning results, in order to improve the effect of tennis teaching.

As can be seen from Figures 1 and 2, in college physical education, the demand for tennis courses increases year by year, while the actual course supply decreases year by year. There is a balance between demand and supply in 2015, and the gap will increase from 2015 to 2020. Therefore, tennis teaching has great potential and needs to be solved more accurately.

## 2. Literature Review

There are many research studies on the cloud computing and deep learning model in tennis teaching, but it mainly stays at the theoretical level and lacks practical case studies [4]. Some scholars believed that the increase of tennis content, the application of information technology, and the reduction of teaching time affected the effect of tennis teaching. Some scholars also believed that the intelligent storage student management scale can realize the management of tennis teaching content and can improve the teaching effect of tennis [5]. Some scholars believed that students' classification and achievement integration can improve students' potential and realize personalized teaching [6]. Some scholars believed that the integration of teaching theory and practice and the division of grades can improve the effect of classroom teaching [7]. Some scholars also believed that the intelligent score management scale, score grade, and potential development were the indicators for the evaluation of tennis teaching effect [8], which can realize the comprehensive analysis of students and tennis teaching. In conclusion, scholars at home and abroad believed that the student intelligent score management scale and cloud computing and deep learning method can improve the teaching effect, realize the integration of students' potential and teaching requirements, and meet the requirements of quality education [9]. However, there was a lack of practical case analysis at home and abroad. On this basis, this paper integrates theory and practice to analyze the effect of cloud computing and deep learning [10].

## 3. Research Model

### 3.1. Cloud Computing and Deep Learning Theory

Cloud computing and deep learning can meet the complex needs of students' learning and is composed of multiple management units. Cloud computing and deep learning can realize the “personalized service” of students and the resource sharing of tennis teaching [11]. First, the tennis teaching scheme is used to divide the “virtual file” for students in the tennis course management center. Then, a management table is built and stored in each student's client node l to form a small-scale data search [12]. Finally, any client node _*l*_ calculates the management table of adjacent clients (node *l* + 1, node *l* − 1) to find the required teaching effect data and return the key value of the corresponding client, node_*i*_⇄_DiskTracker_*i*_(ID_*j*_)*IP*_*k*__^keyvalue^datacenter.

### 3.2. Basic Theory of Cloud Computing and Deep Learning

It is based on the multivariate difference equation, and its mathematical expression is as follows:

(1) $$\begin{array}{c} \left\{\begin{array}{c} {\text{node}}_{l}=A\cdot {\text{DiskTracker}}_{i}+B\cdot {\text{ID}}_{j}+C\cdot {\text{IP}}_{k},\\ {\text{keyvalue}}_{j}=D\cdot {\text{DiskTracker}}_{i}+E\cdot {\text{ID}}_{j}+F\cdot {\text{IP}}_{k}+p\;\sin\left(2k\pi \left(f_{e}+\frac{f_{D}}{f_{s}}\right)\right)\times T\left(k\right). \end{array}\right) \end{array}$$

Among them, A, B, C, and D are the coefficient values of corresponding parameters in tennis teaching; *f*_*e*_, *f*_*s*_, and *f*_*D*_ are the collected data, sent data, and feedback data; *P* is the data amplification factor, which aims to improve the data recognition rate of “abnormal students,” and *T*(*k*) is the data actually received by the center. According to the results of *f*_*e*_, *f*_*s*_, and *f*_*D*_, the level of students' tennis teaching is judged. If *f*_*e*_=*f*_*s*_=*f*_*D*_ ≠ 0 students' tennis teaching is normal, and if *f*_*s*_ ≠ *f*_*D*_=0 is near the extreme value, it indicates that students' tennis teaching is abnormal [13].

### 3.3. Cloud Computing and Deep Learning Process in Tennis Teaching

(1) Data access to students' teaching archives. The access process to students' teaching archive data can be described by a nonlinear Lagrange equation [14], and the mathematical formula is as follows:
  (2) $$\begin{array}{c} g=\frac{d{\text{DiskTracker}}_{i}}{d{\text{node}}_{l}}=-v^{\prime }\left({\text{DiskTracker}}_{i}\right)+F_{0}+g\left({\text{node}}_{l}\right). \end{array}$$
Among them, *g*(node_*l*_) is the gap between students' academic achievements; *F*_0_ represents the collection amount of student effect data; *F*_0_ is a nonlinear discrete function, which *v*′(DiskTracker_*i*_) is the sharing of teaching resources and the satisfaction of individual needs.
(2) Adjustment of the number of student files. The adjustment of the number of student files is a key factor in the cloud computing and deep learning level, which determines the degree of tennis teaching pressure, and its mathematical calculation formula is as follows:
  (3) $$\begin{array}{c} E\left[g\left({\text{node}}_{l}\right)g\left({\text{node}}_{l}+\alpha \right)\right]=6Kg\left({\text{node}}_{l}-\alpha \right)+\xi , \end{array}$$
where *K* is the frequency of tennis resource acquisition; *ξ* is the error value of tennis learning achievement change; *E* is the adjustment coefficient of the total number of students [15].
(3) Effective data transmission. The effective data transmission *F*_0_ determines the level of tennis teaching, and its mathematical calculation formula is as follows:
  (4) $$\begin{array}{c} F_{0}=A_{0}\;\cos\left(2\pi f_{0}{\text{node}}_{l}\right). \end{array}$$
Among them, *A*_0_ is the function amplitude of students' achievement change, and *f*_0_ is the frequency of teaching, which together determine the amount of tennis teaching; teaching effect grade = actual assessment result/expected teaching result*∗*100%.
(4) Shared and personalized service satisfaction. Cloud computing and deep learning requires to evaluate students' tennis learning effect and meet the sharing of public resources and the satisfaction of individual resources [16], which *v*′(DiskTracker)_*i*_ is expressed by a function, and its mathematical calculation formula is as follows:
  (5) $$\begin{array}{c} v^{\prime }\left({\text{DiskTracker}}_{i}\right)=\frac{m}{m+n}f_{g}{\left({\text{DiskTracker}}_{i}\right)}^{2}\\ +\frac{n}{m+n}f_{h}{\left({\text{DiskTracker}}_{i}\right)}^{4}, \end{array}$$
where *m* and *n* are the proportion of shared resources and individual needs in the virtual file, respectively; *f*_*g*_ and *f*_*h*_ are a resource sharing function and personality satisfaction function, both of which are internal algorithms in the tennis teaching scheme [17].
(5) Judgment of critical value. By deriving formula (5), its inflection point can be obtained, that is
  (6) $$\begin{array}{c} v^{\prime \prime }\left({\text{DiskTracker}}_{i}\right)=2\frac{m}{m+n}f_{g}^{\prime }\left({\text{DiskTracker}}_{i}\right)\\ +4\frac{n}{m+n}f_{h}^{\prime }\left({\text{DiskTracker}}_{i}\right). \end{array}$$
After substituting formula (4), it shows that the proportion of shared resources and personalized service resources is in a two-way balance, that is $A_{0}<\sqrt{4m^{2}+mn/27n\left(m+n\right)}$, and the proportion between tennis teaching requirements and actual tennis teaching is the best. In order to better analyze the effect of students' tennis teaching, it will be limited to [−$\sqrt{4m^{2}+mn/27n\left(m+n\right)}$].
(6) Identification of abnormal students. The amplification factor is *λ*, which is added in tennis teaching to identify the abnormal changes of academic performance. If there is a significant change in the scores of any students in the process of tennis teaching, it indicates that the relationship between tennis teaching and students' learning is normal teaching, otherwise, it is students' abnormal learning, and the corresponding data are amplified to identify abnormal students.

### 3.4. Constraints of Cloud Computing and Deep Learning Model

In the cloud computing and deep learning of tennis teaching, the original tennis teaching management method is too simple, leaving the analysis of shared resources and personalized service resources to teachers, increasing the work pressure of teachers, and reducing the management level of students Martins et al. [18]. In view of the above problems, this paper introduces to jointly optimize tennis teaching management and transfer the analysis of some students' teaching to students.

Firstly, metropolis constraint, this paper uses metropolis constraints to judge the effectiveness of student information, so as to reduce the impact of invalid information on the results. If the result is “0,” it indicates that the data is invalid, eliminated, or the value is enlarged, otherwise, the corresponding calculation is conducted. After the data is constrained by metropolis, a value is assigned to it to make the constraint result “0” or “1,” and the standardization process is completed. According to the above analysis, the mathematical conditions are as follows:

(7) $$\begin{array}{c} \left\{\begin{array}{c} {\text{keyvalue}}_{j}\neq {\text{keyvalue}}_{j+1}\neq 0,\\ {\text{keyvalue}}_{j}={\text{keyvalue}}_{j+1},{\text{keyvalue}}_{j}\neq 0, \end{array}\right) \end{array}$$

where *M*(*·*) is the judgment function of metropolis constraint.

Secondly, the matching between actual teaching and expected teaching effect. The matching between the actual teaching and the expected teaching effect is complex and multidimensional. The actual teaching effect of tennis is not only affected by the number of students but also by the requirements of “sharing degree” and “personality degree.” Assuming that the matching of “sharing degree” is *P*_*u*_ and the matching of “personality degree” is *P*_*v*_, formula (5) can be optimized as follows:

(8) $$\begin{array}{c} P=\left\{\begin{array}{c} \prod \left[\sum_{i}^{\infty }v^{\prime }\left({\text{DiskTracker}}_{i}\right)+\varsigma \right],\\ \frac{\kappa \left(P_{u}-P_{\min}\right)}{P_{\max}-P_{\min},P_{u}<P_{v}},\\ \frac{\lambda \left(P_{v}-P_{\min}\right)}{P_{\max}-P_{\min},P_{v}<p_{u}}, \end{array}\right) \end{array}$$

where *P*_max_ and *P*_min_ are the maximum and minimum bearing matching values of tennis teaching, the adjustment coefficient of personalized matching, and the matching coefficient of sharing degree.

Thirdly, the effective evaluation and student volume of cloud computing and deep learning. In order to reduce the overload impact of teaching time on tennis teaching, a part of the analysis of teaching effect is analyzed by students, and the management table is introduced to judge the degree of teaching sharing. The original formulas (2) and (3) are optimized into the following formulas:

(9) $$\begin{array}{c} \left\{\begin{array}{c} R=\int_{i,j}^{n}\begin{array}{c} \sum_{l}^{\infty }\lim g\left({\text{node}}_{l}\right)\left[-v^{\prime }\left({\text{DiskTracker}}_{i}\right)\right]+H_{i}\cdot f\left(\hat{{\text{DiskTracker}}_{i}},\hat{{\text{node}}_{l}}\right),\;R=1, \end{array}\\ U=\int_{i,j}^{n}\left(\sum_{l}^{\infty }\lim g\left({\text{node}}_{l}\right)\right]\left\{\begin{array}{c} E\left[g\left({\text{node}}_{l}\right)\right]++H_{i}\cdot f\left(\hat{{\text{node}}_{l}},\hat{g\left({\text{node}}_{l}\right)}\right) \end{array}\right\}, \end{array}\right) \end{array}$$

where R is the number of visits to teaching resources, and its value is 0, indicating that teaching resources are not accessed, and students can use the management list to search resources among students; *U* is the number of user visits. The number of students in the preset time is compared with the maximum standard required by tennis teaching. If the ratio is > 9/10, it indicates that the effect of network teaching is good, and the research is strengthened on corresponding teaching contents; $f\left(\hat{{\text{node}}_{l}},\hat{g\left({\text{node}}_{l}\right)}\right)$ is the calculation function of students' misunderstanding rate in tennis delivery; *H*_*i*_ is the adjustment coefficient of misunderstanding. The judgment process is shown in Figure 3.

Fourthly, the construction steps of cloud computing and deep learning optimization model. According to the student learning scale and the data description formula of tennis teaching, the simulation model is built. The specific steps are as follows:

1. In the cloud computing and deep learning scale, the more frequent the intragroup teaching visits between students through the management scale, the less the pressure of actual tennis teaching and the higher the tennis teaching effect. Therefore, node_*i*_⇄_DiskTracker_*i*_(*ID*_*j*_)*IP*_*k*__^keyvalue^datacenter is the best critical value required first, and this value is taken as the stable threshold of the whole tennis teaching. The result of the threshold must be in [−$\sqrt{m^{2}+mn/n\left(m+n\right)}$, $\sqrt{4m^{2}+mn/27n\left(m+n\right)}$].
2. Identifying abnormal students in tennis teaching. The abnormality of data transmission in cloud computing and deep learning is an important optimization index. The occurrence of abnormal data is determined by many factors, such as the management table, the integration of DHT and tennis teaching scheme, the division of virtual space in tennis teaching, field type, byte size, access time, and system load. Under the constraint of keyvalue_*j*_ ≠ keyvalue_*j*+1_ ≠ 0, $A_{0}<\sqrt{4m^{2}+mn/27n\left(m+n\right)}$ is the data transmission relatively stable, and the data transmission between tennis teaching and cloud computing and deep learning is normal.
3. Building a simulation model of tennis teaching effect. The teaching effect is the final result of tennis teaching and students' understanding, and is affected by the requirements of quality education, teaching time, teaching methods (multimedia, online, and offline), as well as students' own interests. The actual effect of tennis teaching is consistent with the expected requirements, indicating that the effect of tennis teaching meets the requirements. Among them, the calculation of teaching effect is divided into shared resource teaching *P*_*u*_ and personalized service teaching *P*_*v*_. In the calculation process, the number of visits *R* and *U* of students is checked in the virtual file, and the consistency between the teaching level and the teaching requirements is judged.

## 4. Case Analysis of Cloud Computing and Deep Learning Model on Tennis Teaching Effect Evaluation

### 4.1. Case Introduction

Taking the 48 h tennis teaching course of a university as an example, 32 classes of offline students are managed. Tennis teaching evaluation needs 1 server, 4 PCs, and 12 mobile phones. The storage mode of students' virtual archives is the combination of disk and solid state, and the storage space is 723 t. The specific circuit diagram is shown in Figure 3. Each student carries out wireless communication through the terminal and sets up their own LAN. Teachers accept students' real-time data and historical data. The data interfaces are filtered signal interface, setting out signal interface, AD conversion interface, and data metering port.

### 4.2. Judgment and Comparison of Tennis Teaching Results by Cloud Computing and Deep Learning

The model built by Simulink in MATLAB software is used for analysis, and the results are shown in Figure 4. Firstly, the data fit. In the cloud computing and deep learning of tennis teaching, the fitting degree between actual teaching and expected teaching is an important management evaluation index. The results are shown in Figure 4.

It can be seen from Figure 4 that the simulation of intelligent teaching is carried out by using a time timer and input waveform device; the maximum value, intermediate value, and minimum value are analyzed. Among them, the matching rate between the actual teaching data and the expectation is shown in Figure 5.

It can be seen from Figure 5 that the expected evaluation requirements of intelligent teaching are basically consistent with the actual requirements, indicating that the constructed simulation model can analyze cloud computing and deep learning. In short, the simulation model constructed in this paper is effective and can be used for practical case analysis. It can be seen from Figures 4 and 5 that the fitting degree *p* between the actual teaching and the expected teaching requirements is good. The reason is that before judging, the tennis teaching effects are carried out, and the amplification factor *p* in the management table is used to identify abnormal students and take targeted teaching and training. In addition, the teaching data in Figure 6 is relatively stable and the slope changes less. At the same time, the change range of the actual teaching data is relatively stable, which shows that the data processing of the actual teaching is relatively stable, which further shows the effectiveness of the algorithm. The reason is that the “group” built by students themselves and the sharing of tennis teaching resources can realize students' autonomous learning and more efficient understanding of tennis content, and continuously improve their own knowledge combined with offline teaching content.

Secondly, the level of tennis teaching effect. Tennis teaching level is the focus of cloud computing and deep learning, which involves the content of practical operation and theoretical students. Compared with the traditional centralized mode, cloud computing and deep learning mode has a higher level of teaching effect. On the whole, the evaluation data of actual teaching effect changes little, and the overall comparison process meets the evaluation requirements of learning effect. The reason is due to the self-help learning among students and the effective utilization of teaching resources. The results are shown in Figure 7.

As can be seen from Figure 7, the teaching level under the cloud computing and deep learning method is higher, and the teaching level is also higher than the original evaluation method. At the same time, the fluctuation range of the two algorithms is different. The fluctuation range of the algorithm proposed in this paper is small and meets the requirements of teaching effect evaluation. The comparison of teaching levels of different methods is shown in Figure 8.

As can be seen from Figure 8, the cloud computing and deep learning method is higher than the original management method in terms of personalized service/resource. Compared with the original method, the algorithm proposed in this paper can evaluate the teaching effect more effectively. The main reason is the horizontal analysis of cloud computing and the vertical analysis of deep learning so as to realize the comprehensive judgment of the effect of intelligent teaching. The comparison of the personalized service/resource sharing ratio of different methods is shown in Figure 9.

As can be seen from Figures 9 and 10 that the calculation results of the two algorithms are higher in terms of service and resource sharing. Compared with the original method, the algorithm proposed in this paper mainly focuses on the core area of the radiograph. Therefore, the personalized strategy and resource sharing of the algorithm proposed in this paper are better than the original algorithm sharing ratio. This shows that under the same teaching time, the cloud computing and deep learning method can provide a higher proportion of personalized services. As we all know, personalized service is one of the important contents of quality education. The cloud computing and deep learning method improves the processing efficiency of tennis teaching on relevant teaching contents and reduces tennis teaching time according to the optimization methods such as the management table so as to better provide personalized management services to students.

## 5. Conclusion

Cloud computing and deep learning can evaluate the effect of tennis teaching in colleges and universities [19]. Cloud computing and deep learning can make up for the deficiency of single teaching and improve the accuracy of tennis teaching effect evaluation. At the same time, cloud computing and deep learning can shorten the evaluation time of teaching effect and make tennis teaching better meet the intelligent requirements. Cloud computing and deep learning is a management method based on middle school teaching. This method comprehensively evaluates the tennis teaching effect by preprocessing the tennis teaching evaluation data so that the evaluation results are more in line with the actual requirements. Cloud computing and deep learning methods reduce the amount of preprocessed data and evaluate the effect faster by identifying “abnormal data.” MATLAB simulation results show that under cloud computing and deep learning, the fitting degree *p* between the actual tennis teaching effect and the expected teaching effect is better, and the tennis teaching effect level and the ratio of personalized service/resource sharing are higher than the original teaching method. Therefore, in the case of limited teaching time and complex teaching content, the cloud computing and deep learning method can effectively improve the tennis teaching effect and realize the personalized training of students.

## Figures and Tables

**Figure 1:** Changes in tennis teaching hours.

**Figure 2:** The supply and demand of tennis courses.

**Figure 3:** The judgment process of tennis courses.

**Figure 4:** The cloud computing and deep learning simulation of college tennis teaching.

**Figure 5:** The fit ratio of data transmission between actual teaching and expected teaching requirements.

**Figure 6:** The changes in actual teaching data.

**Figure 7:** The comparison between cloud computing and deep learning and the original management method.

**Figure 8:** The comparison of teaching effect levels of different methods.

**Figure 9:** The personalized service/resource sharing ratio of the two algorithms.

**Figure 10:** The improvement degree of teaching effect of the two algorithms.

## Data Availability

The data used to support the findings of this study are available from the corresponding author upon request.
